The article "Application and Evaluation of a 64-Slice CT Three-Dimensional Fusion Technique in the Determination of the Effective Ablation Margin after Radiofrequency Ablation of Hepatocellular Carcinoma" was retracted in 2023. Reasons: unreliable results or conclusions; concerns about the data; concerns about the peer review; concerns about the citations.

# Application and Evaluation of a 64-Slice CT Three-Dimensional Fusion Technique in the Determination of the Effective Ablation Margin after Radiofrequency Ablation of Hepatocellular Carcinoma

**DOI:** 10.1155/2022/6898233

**Published:** 2022-01-27

**Authors:** Haihao Du, Xiongmu Tan, Liuhui Cheng, Baopeng Zhang, Daoqing Wang

**Affiliations:** ^1^Department of Radiology, The First Affiliated Hospital of Henan University of CM, Zhengzhou, Henan 450000, China; ^2^Department of Radiology, Sichuan Cancer Hospital, Chengdu, Sichuan 640041, China

## Abstract

Due to the low accuracy of traditional three-dimensional fusion technology in radiofrequency ablation of hepatocellular carcinoma, this paper studies the advantages of three-dimensional CT fusion technology over traditional two-dimensional imaging technology in preoperative visualization and radiofrequency ablation path selection of hepatocellular carcinoma. To study the prognostic differences of hepatocellular carcinoma patients with different ablation margins (AM) in the three groups, so as to explore the best AM value, so as to minimize the liver injury caused by radiofrequency ablation. The selected patients underwent CT plain scan and three-phase enhancement at 1, 3, 6, and 12 months after operation and were rechecked every 6 months. For recurrent patients, CT was rechecked every three months. The images were obtained by GE 64-slice spiral CT. The thickness of the reconstruction layer is 1 mm, and the interval is 1 mm. The reconstructed image is imported into 3D fusion software. The three-dimensional images of tumor focus, hepatic artery, portal vein, and hepatic vein were reconstructed by two experienced doctors by superimposing the saved tumor images, merging the vascular images into the display, and measuring the ablation boundary (AM value). The results showed that the recurrence rate in group A was higher than that in group B (*P* = 0.041), and there was no significant difference between group B and group C (*P* = 1.000). Compared with traditional two-dimensional imaging, three-dimensional CT fusion technology can display the anatomical structure and three-dimensional spatial relationship of tumors and blood vessels and select the best radiofrequency ablation path, so as to achieve accurate radiofrequency ablation.

## 1. Introduction

Primary liver cancer (HCC) is one of the most common malignant tumors in the world and has the third-highest mortality among malignant tumors [1–4]. In China, the HCC incidence and mortality are particularly high. There are 400 000 new liver cancer diagnoses in China every year, and this number appears to be increasing [5–7]. Most patients with liver cancer progress from hepatitis to cirrhosis to liver cancer, a process that may take between 10 and 20 years. Studies [8–11] have shown that the larger the HCC diameter, the greater the probability of metastasis, microvascular invasion, and satellite focus and the worse the patient's prognosis. Therefore, early treatment of small hepatocellular carcinoma (SHCC) can greatly improve the patient's prognosis, quality of life, and survival rate.

The article "Application and Evaluation of a 64-Slice CT Three-Dimensional Fusion Technique in the Determination of the Effective Ablation Margin after Radiofrequency Ablation of Hepatocellular Carcinoma" was retracted in 2023. Reasons: unreliable results or conclusions; concerns about the data; concerns about the peer review; concerns about the citations.

Radiofrequency ablation includes inserting a radiofrequency needle into the tumor under imaging guidance; RF current is emitted through the microelectrode, which causes the vibration of charged ions in the tissue, quickly generates heat, and leads to coagulative necrosis of cells around the electrode. RFA has the advantages of safety, minimally invasive, less complications, short hospital stay, less surgical pain, rapid recovery, and repeatable treatment. It is the most promising minimally invasive treatment for SHCC and is also accepted by most patients. For SHCC ≤ 3 cm in diameter, there was no significant difference between RFA and surgical prognosis [12, 13]. Although some SHCC can be completely cured by RFA, RFA cannot completely remove the tumor due to the irregular growth boundary of the tumor, resulting in a high recurrence rate that is difficult to control. At present, the main factors affecting the efficacy of RFA in the treatment of liver cancer include excessive tumor volume (>3 cm), irregular tumor edge, RF boundary, heat dissipation of adjacent large blood vessels, and liver function. These factors may lead to tumor residue and recurrence [14–17]. There is no clear conclusion about the ideal thickness of ablation edge (AM) formed around the original tumor to make the tumor completely necrotic. Routine clinical aim is 5-10 mm, but further research is needed to determine specific AM values. Therefore, it is necessary to accurately measure the RF boundary after treatment, accurately judge the degree and scope of necrosis, prevent postoperative recurrence, ensure the integrity of treatment, and improve the survival rate of patients.

At present, traditional imaging methods are used to evaluate the size, boundary, and potential postoperative prognosis before RFA treatment. However, they cannot observe the tumor volume, boundary, and ablation of the cancer directly and stereoscopically after RFA. The complexity of the hepatic vascular system, the compression of the tumor itself, and irregularity of the growth boundary make RFA treatment more difficult while damage to the hepatic vascular system can easily occur. Traditional two-dimensional CT cannot display both the anatomical structure of the liver, tumor, and vascular system and their three-dimensional spatial relationships. With the development of medical imaging technology, three-dimensional fusion reconstruction technology has emerged to meet these requirements. The combination of modern medical imaging and three-dimensional fusion technology allows accurate preoperative evaluation and prediction of the postoperative effects of RFA, thus spanning research in many disciplines.

The article "Application and Evaluation of a 64-Slice CT Three-Dimensional Fusion Technique in the Determination of the Effective Ablation Margin after Radiofrequency Ablation of Hepatocellular Carcinoma" was retracted in 2023. Reasons: unreliable results or conclusions; concerns about the data; concerns about the peer review; concerns about the citations.

## 2. Methods

### 2.1. Research Subjects

Thirty-one patients with 42 primary liver cancer lesions were selected in the First Affiliated Hospital of Henan University of Traditional Chinese Medicine from January 2016 to September 2018. The range of the maximum axial diameter of the tumor was 8.2-44.4 mm. The patients included 19 men and 12 women with an average age of 51 ± 12.3 years ranging from 34 to 76 years. According to the Child-Pugh liver function classification, there were 20 cases of grade A and 11 cases of grade B. Of the 31 patients, 90.3% (28/31) had a history of hepatitis while 71.0% (22/31) had a history of liver cirrhosis. All tumors were clinically confirmed as primary liver cancer. All patients signed informed consent.

### 2.2. Inclusion Criteria

1. Primary hepatocellular carcinoma was confirmed by pathological biopsy or clinical diagnosis
2. The diameter of the tumor was less than or equal to 5 cm
3. There was no vascular tumor thrombus and adjacent organ invasion
4. The imaging findings were typical of primary liver cancer
5. The patient was in good condition, without obvious organic lesions of the heart, lung, kidney, and other important organs, and the function was in good condition or only slightly damaged
6. Liver function is of A or B grade according to the liver function classification

### 2.3. Exclusion Criteria

1. The distance between tumor and blood vessel was less than 0.5 cm
2. The presence of uncorrectable coagulation dysfunction and tendency for severe bleeding
3. Intractable massive ascites
4. Patients with mental disorders or who were unable to cooperate with the treatment
5. Patients with hyperthyroidism, history of iodine contrast agent allergy, severe heart, liver, or kidney dysfunction, pregnancy, or bronchial asthma

## 3. Acquisition of CT Images

In the scanning room, the patient lay flat on the scanning table with both arms raised. The transverse positioning line was about two transverse fingers on the upper edge of the sternal angle, and the bilateral positioning lines coincided with the axillary midline. The double-barrel high-pressure syringe and the patient's indwelling needle were connected, injecting normal saline to ensure that the enhanced contrast agent could enter the patient's body unobstructed during the enhanced scanning. The upper abdominal plain scan image was obtained first, with a scanning range from the septum to the lower edge of the liver (in some patients with liver cirrhosis, the spleen was larger than the lower edge of the liver, so the spleen should be included in the scan). The parameters of upper abdomen continuous CT scanning included voltage 120 kV, current 250 Ma, collimation 64 × 0.625 mm, slice thickness 5 mm, and spacing 5 mm. The contrast medium was injected through the median cubital vein with a high-pressure syringe with an injection speed of 4.5 ml/s. The contrast medium was Omnipaque (iohexol) with a concentration of 350 mgI/ml. The scanning range and parameters were the same as those of the plain scan. The delay times of the hepatic artery, portal vein, and equilibrium phases were 25-30 s, 55-60 s, and 80-90 s, respectively (180 s delay scan can be performed if delay scan is needed). At the end of the scan, the four-phase images of the upper abdomen were obtained, including the plain scan, arterial, portal, and equilibrium phases. The four-phase images were reconstructed with a thickness of 1 mm and an interval of 1 mm, and the reconstructed thin-layer images were stored in the CT postprocessing workstation.

The article "Application and Evaluation of a 64-Slice CT Three-Dimensional Fusion Technique in the Determination of the Effective Ablation Margin after Radiofrequency Ablation of Hepatocellular Carcinoma" was retracted in 2023. Reasons: unreliable results or conclusions; concerns about the data; concerns about the peer review; concerns about the citations.

### 3.1. The Three-Dimensional Fusion Reconstruction Steps

The reconstructed four-phase thin-layer images were transferred from the CT postprocessing workstation to the GE postprocessing software, and the volume rendering (VR) mode was selected. The arterial phase was used to reconstruct the tumor, selecting auto select and any in turn structure button, moving the mouse to the location of the lesion and clicking, thus automatically drawing the boundary of the tumor. However, due to the irregular shape of the tumor growth, the accuracy of automatic recognition is insufficient and manual modulation and addition are needed. The tumor was generally drawn through the axial image at each level from the first level where the tumor was visible to the last where it was no longer visible. After sketching all the tumor layers, the image was saved using “save volume” (if the tumor was not clearly displayed, the middle mouse button could be dragged back and forth until a satisfactory image was displayed), completing the three-dimensional imaging of the tumor. For the reconstruction of the intrahepatic vascular system (including the hepatic artery, portal vein, and hepatic vein), the hepatic artery was reconstructed using the arterial phase, selecting “auto select, any” and clicking the “structure” button, and moving the mouse to the root of the hepatic artery, allowing the hepatic artery to be automatically identified. If the contrast agent filling in the hepatic artery is not good, the hepatic artery can be manually added using the axial image and can be cut if necessary. After all layers are added and cut, the image is saved. The three-dimensional imaging steps of the portal and hepatic veins were the same as those of the hepatic artery, calling out the saved three-dimensional images of the tumor focus, hepatic artery, portal and hepatic veins, selecting the VR mode, and clicking the image “multi.” The hepatic artery, portal vein, and hepatic vein are then dragged into the display screen where the tumor is located to complete the three-dimensional fusion reconstruction of the tumor and intrahepatic vascular system. Finally, the “save state” function is clicked to save the fused three-dimensional state image.

The article "Application and Evaluation of a 64-Slice CT Three-Dimensional Fusion Technique in the Determination of the Effective Ablation Margin after Radiofrequency Ablation of Hepatocellular Carcinoma" was retracted in 2023. Reasons: unreliable results or conclusions; concerns about the data; concerns about the peer review; concerns about the citations.

### 3.2. Selection of Reference Materials and Data Measurement of Tumor and Ablation Focus before and after RFA Treatment

1. For the selection of reference materials for the tumor and its ablation before and after RFA treatment, the reconstructed four-phase thin-layer images were transferred to the CT reader, the reference materials were selected according to the specific location of the tumor, and the diameter of the tumor was measured. As the liver moved up and down with human breathing, the reference materials could be selected in the liver as much as possible. In this study, 42 tumor foci were selected as reference materials including 40 liver capsule and 2 portal vein branches
2. Measurement of tumor and ablation data before and after RFA treatment involved calling out the axial images of the tumor and ablation before and after RFA treatment and measuring the data under the guidance of two experienced doctors. The maximum axial section of the tumor or ablation focus was first identified and the maximum cross section measured, recording the data. The reference was selected (the references selected before and after ablation should be consistent), and the distance from the reference to the boundary of the tumor or ablation focus on the maximum cross section measured, followed by selection of the reference its measurement to the tumor or ablation focus on the upper and lower levels (depending on the size of the tumor). If the distance between the liver capsule and the tumor is less than or equal to 1 cm, the distance from the reference object passing through the center of the tumor to the contralateral edge is measured as the ablation range is larger than that of the tumor during radiofrequency ablation. If the distance between the liver capsule and the tumor is small, it cannot be measured after radiofrequency ablation. The measurements are conducted on the axial image as the data measured on the axial image is the most accurate and convincing
3. The size of the ablation boundary was calculated by subtracting the data measured before RFA from the data measured after RFA. The patients were divided into three groups according to the size of the ablation boundary: group A: AM greater than or equal to 5 mm but less than 8 mm; group B: AM greater than or equal to 8 mm but less than 10 mm; group C: AM greater than or equal to 10 mm

The article "Application and Evaluation of a 64-Slice CT Three-Dimensional Fusion Technique in the Determination of the Effective Ablation Margin after Radiofrequency Ablation of Hepatocellular Carcinoma" was retracted in 2023. Reasons: unreliable results or conclusions; concerns about the data; concerns about the peer review; concerns about the citations.

### 3.3. Postoperative Follow-Up

All patients were followed up regularly. CT plain scans and three-phase enhanced scans were performed at 1, 3, 6, and 12 months after the operation, and the CT was reexamined every six months. For patients with recurrence, CT was reexamined every three months. At the same time, combined with clinical examination, the indices of alpha-fetoprotein (AFP), liver function, and coagulation function were reexamined.

### 3.4. Criteria for Imaging Evaluation of Recurrence

Complete ablation: early examination showed that the ablation area was larger than the preoperative area. At follow-up, the ablation area volume became gradually smaller. There was no obvious enhancement in the arterial phase, and the boundaries of the lesions were clear in the portal and equilibrium phases.

Incomplete ablation: the ablation area was not significantly reduced; there were irregular enhancement bands at the edge with weakened enhancement in the portal and equilibrium phases, with this type of enhancement present in later reviews. Alternatively, although the ablation area was reduced in the continuous follow-up, circular and quasicircular enhancement was visible in the enhanced scan, with the degree of enhancement decreasing in the portal and equilibrium phases, with the characteristic of “fast in and fast out.”

## 4. Results

### 4.1. Clinical Data Analysis

Of the 31 patients, comprising 42 lesions, 19 were male and 12 were female. The age of patients ranged from 34 to 76 years old. The average age of patients was 51.1 ± 12.3 years old. According to the Child-Pugh liver function classification, there were 20 cases of grade A and 11 cases of grade B. Of the 31 patients, 90.3% (28/31) had a history of hepatitis and 71.0% (22/31) had a history of liver cirrhosis. The maximum axial diameter of the tumors ranged between 8.2 and 44.4 mm. The analysis of the clinical data is shown in Table 1.

According to Table 1, the pathological conditions of patients in groups A, B, and C can be fully understood. According to the results of statistical methods, *P* < 0.05, no significant difference, and no influence on later experiments.

### 4.2. AM Measurements after RFA

After RFA, the patients were divided into three groups according to the size of the AM: group A, AM greater than or equal to 5 mm but less than 8 mm; group B, AM greater than or equal to 8 mm but less than 10 mm; and group C, AM greater than or equal to 10 mm. In order to evaluate the effect of different AMs on postoperative recurrence, we compared the postoperative recurrence rate of each group. The recurrence rate data of each group are shown in Table 2 and Figure 1.

The article "Application and Evaluation of a 64-Slice CT Three-Dimensional Fusion Technique in the Determination of the Effective Ablation Margin after Radiofrequency Ablation of Hepatocellular Carcinoma" was retracted in 2023. Reasons: unreliable results or conclusions; concerns about the data; concerns about the peer review; concerns about the citations.

According to the data in Table 2 and Figure 1, the overall recurrence rate was 43.75%, while that in group A was 6.25%, 12.5%, 25%, 37.5%, and 43.75% at 6, 12, 18, 24, and 30 months after, respectively; in group B, 0, 6.25%, 6.25%, 6.25%, and 6.25% for 6, 12, 18, 24, and 30 months; and in group C, 0, 0, 10%, 10%, and 10% at 6, 12, 18,24, and 30 months after the operation, respectively. In order to compare the postoperative recurrence rate of RFA in different AMs, we compared the three groups. It was found that the recurrence rate in group A was higher than that in group B and group C. There was no significant difference between group B and group C, but there was a significant difference compared with group A. The schematic diagram of CT image acquisition is shown in Figures 2–7.

## 5. Discussion

With the development of imaging technology, the measurement of radiofrequency ablation boundary has made some progress. Ahn et al. [18] prospectively discussed the feasibility and prognosis of real-time ultrasound MRI-CT image fusion technology in radiofrequency ablation of liver cancer. The effectiveness and visibility of fusion imaging-guided radiofrequency ablation are similar to those of conventional ultrasound guidance, and ultrasound-CT-MRI combined with fusion imaging guidance can improve the visibility of tumor and the feasibility of radiofrequency ablation in patients with liver cancer.

In addition, fusion imaging-guided multielectrode radiofrequency ablation showed higher technical efficiency and lower local tumor progression rate in midterm follow-up. Kai et al. [19] proved that 3D ultrasound CT image fusion has high accuracy in evaluating the safety boundary of liver cancer in vitro, but it needs to be further explored in human 3D ultrasound CT fusion. Makino et al. [20] observed the effect of radiofrequency ablation in 94 patients with liver cancer using automatic CT image fusion technology. These authors automatically superimposed and compared CT images before and after RFA to measure the minimum ablation edge (MAM) and evaluate whether it is related to local tumor recurrence. The results show that compared with conventional CT, automatic CT image fusion technology can accurately predict the efficacy of RFA and show the existence of residual tumors after RFA through the quantitative value of man. Tang et al. [21] evaluated 75 patients with small hepatocellular carcinoma before and after radiofrequency ablation with three-dimensional CT image fusion. The results showed that AM was an independent factor after radiofrequency ablation of liver cancer. Conclusion: 3D-CT image fusion technology is a feasible and useful method for accurate measurement and prognosis prediction of an after radiofrequency ablation of liver cancer [22–24]. Jiang et al. [25–27] used three-dimensional reconstruction technology to measure AM in different directions of 159 liver cancer lesions in 134 patients, analyzed the relationship between accurate ablation boundary and local tumor after radiofrequency ablation, and considered that three-dimensional reconstruction technology is a method to accurately evaluate the boundary after radiofrequency ablation [28].

The article "Application and Evaluation of a 64-Slice CT Three-Dimensional Fusion Technique in the Determination of the Effective Ablation Margin after Radiofrequency Ablation of Hepatocellular Carcinoma" was retracted in 2023. Reasons: unreliable results or conclusions; concerns about the data; concerns about the peer review; concerns about the citations.

In this study, AM was calculated by measuring the distance from the reference point before and after RFA to the tumor. The use of in vivo and extrahepatic reference materials (such as vertebral bodies, ribs, sternum, and other anatomical structures) may lead to measurement errors in RFA due to the influence of patient respiratory movement, different patient examination positions, and other extrahepatic reference materials. Because the measurement error before and after RFA may be relatively large [29], this method is rarely used in actual measurement. In this study, we basically selected all intrahepatic reference materials, including hepatic capsule, portal vein and branches of hepatic vein, small calcification of intrahepatic cyst, and other intrahepatic structures. Their fixed position is not easy to change. They move with the movement of breathing and posture [30]. Therefore, the tumor focus and the reference material are in a relatively static state, which ensures that the level measured before and after RFA is at the same level. At the same time, it also ensures the accuracy of measurement before and after RFA [31]. During the measurement, if the distance between the reference and the tumor is less than 1 cm, the distance from the reference to the center of the lesion to the contralateral edge shall be measured. Because the ablation range is larger than the tumor range during RF ablation and the distance between the reference point and the tumor is small, it cannot be measured after RF ablation. Most patients have a history of liver cirrhosis, resulting in uneven and wavy liver edges, which not only increases the difficulty of using the liver capsule as a reference for measurement but also reduces the accuracy of measurement data. Therefore, when selecting the liver capsule as a reference, the smooth or mild cirrhotic edge should be selected.

The article "Application and Evaluation of a 64-Slice CT Three-Dimensional Fusion Technique in the Determination of the Effective Ablation Margin after Radiofrequency Ablation of Hepatocellular Carcinoma" was retracted in 2023. Reasons: unreliable results or conclusions; concerns about the data; concerns about the peer review; concerns about the citations.

## 6. Conclusion

The project combines modern medical imaging with three-dimensional fusion techniques and applies it to preoperative evaluation of RF ablation and postoperative cure prediction across studies in multiple disciplines. In contrast to conventional 2D imaging, CT 3D fusion techniques can show the anatomical structure of tumors and blood vessels and their three-dimensional spatial relationships and innovative in the realization of accurate and accurate RFA treatment by selecting the optimal RF ablation path. By measuring the ablation edges in the preoperative and postoperative images, we can directly and accurately judge the AM, to guide further treatment and accurately determine the prognosis. In this study, we explored the ablation boundary of 8–10 mm. The results suggest that this can achieve good results and could guide clinical ablation of AMs, greater than 8 mm in diameter thereby reducing damage to normal liver tissue.

## Figures and Tables

**Figure 1:** Trend of 30-month recurrence rate in the three groups.

**Figure 2:** Schematic diagram of CT image acquisition. The main tumor is located in the upper part of the right posterior lobe. (a) The tumor diameter before RFA is 44.2 mm. (b) The tumor diameter after RFA is 53.7 mm. (c) The tumor edge recurs 6 months after RFA. (d–g) The spatial relationship between the tumor before RFA and intrahepatic vessels (different color tissues in the figure: red: tumor; yellow: hepatic artery; green: portal vein; purple: hepatic vein and inferior vena cava). The postoperative CT diagram of the patient is shown in Figures 3 and 4.

**Figure 3:** Schematic diagram of postoperative CT. The patient is male. The main tumor is located in the lower part of the right posterior lobe. (a) The diameter of tumor before RFA was 34.6 mm. (b) The diameter of the tumor after RFA was 46.3 mm. (c–f) Spatial relationship between pre-RFA tumor and intrahepatic vessels. No recurrence was found after radiofrequency ablation.

**Figure 4:** Schematic diagram of CT after treatment. The main body of the tumor is located in the upper part of the right anterior lobe. (a) Two-dimensional CT before RFA showed that the tumor diameter was 16.7 mm. (b) Two-dimensional CT. (c–f) After RFA: the spatial relationship between preoperative tumor lesions and intrahepatic vessels. After radiofrequency ablation, there was no recurrence.

**Figure 5:** The main tumor was located in the upper part of the right posterior lobe. (a) Before RFA, the diameter of the tumor was 44.2 mm. (b) After RFA, the diameter of the tumor was 53.7 mm. (c) Six months after RFA, recurrence was found at the edge of the tumor in the upper right posterior lobe. (d–g) The spatial relationship between the tumor and intrahepatic vessels before RFA (tissues represented by various colors in the picture: red: tumor; yellow: hepatic artery; green: portal vein; purple: hepatic vein and inferior vena cava).

The article "Application and Evaluation of a 64-Slice CT Three-Dimensional Fusion Technique in the Determination of the Effective Ablation Margin after Radiofrequency Ablation of Hepatocellular Carcinoma" was retracted in 2023. Reasons: unreliable results or conclusions; concerns about the data; concerns about the peer review; concerns about the citations.

**Figure 6:** The patient was male. The main tumor was located in the lower part of the right posterior lobe. (a) Before RFA, the diameter of the tumor was 34.6 mm. (b) After RFA, the diameter of the tumor was 46.3 mm. (c–f) The spatial relationship between the tumor and intrahepatic vessels before RFA. No recurrence was found after RFA.

**Figure 7:** The main body of the cancer was located in the upper segment of the right anterior lobe. (a) Two-dimensional CT before RFA showed that the diameter of the tumor was 16.7 mm. (b) Two-dimensional CT after RFA. (c–f) Spatial relationship between preoperative cancer focus and intrahepatic vessels in RFA. After RFA, there was no recurrence.

**Table 1:** Clinical and pathological data.

AM size grouping (mm)	Total cases/number of cancer cases (number of cases)	Male/female (number of cases)	Age group (year)	Average median age (year)	History of hepatitis (number of cases)	History of cirrhosis (number of cases)	Child-Pugh liver function classification (number of cases)			AFP level before RFA (number of cases)		
							Level A	Level B	Level C	AFP < 25 ng/ml	25 ng/ml ≤ AFP < 400 ng/ml	AFP ≥ 400 ng/ml
Group A: 5 mm ≤ AM < 8 mm	13/16	8/5	36-76	51.7 ± 14.62	11	7	9	4	0	4	7	2
Group B: 8 mm ≤ AM < 10 mm	11/16	7/4	36-68	53.5 ± 10.21	10	9	6	5	0	2	8	1
Group C: AM ≥ 10 mm	7/10	4/3	34-71	49.3 ± 17.32	7	6	5	2	0	2	3	2
Total	31/42	19/12	34-76	51.1 ± 12.3	28	22	20	11	0	8	18	5

**Table 2:** Comparison of recurrence among the different groups after RF.

	Complete cure after RFA (number of cases)	Recurrence after RFA (number of cases)	*χ* ^2^ value	*P* value
Group A	9	7	6.071	4.375
Group B	15	1	4.167	0.041
Group C	9	1	0.000	1.000

## Data Availability

The data underlying the results presented in the study are available within the manuscript.

## References

[1] Mcglynn K. A., Petrick J. L., London W. T. (2015). Global epidemiology of hepatocellular carcinoma: an emphasis on demographic and regional variability. *Clinics in Liver Disease*.

[2] Mcglynn K. A., Petrick J. L., El-Serag H. B. (2020). *Epidemiology of Hepatocellular Carcinoma*.

[3] Mohamed F. H., Abdallah M. D., Shimaa H. I. (2021). Follow-up after radiofrequency ablation of hepatocellular carcinoma; diffusion weighted & dynamic contrast enhanced MRI characteristics. *The Medical Journal of Cairo University*.

The article "Application and Evaluation of a 64-Slice CT Three-Dimensional Fusion Technique in the Determination of the Effective Ablation Margin after Radiofrequency Ablation of Hepatocellular Carcinoma" was retracted in 2023. Reasons: unreliable results or conclusions; concerns about the data; concerns about the peer review; concerns about the citations.

[4] Global Burden of Disease Cancer Collaboration, Fitzmaurice C., Akinyemiju T. F. (2018). Global, regional, and national cancer incidence, mortality, years of life lost, years lived with disability, and disability-adjusted life-years for 29 cancer groups, 1990 to 2016: a systematic analysis for the Global Burden of Disease study. *Oncologia*.

[5] Chen W., Zheng R., Baade P. D. (2016). Cancer statistics in China, 2015. *CA: a Cancer Journal for Clinicians*.

[6] Cao W., Chen H.-D., Yu Y.-W., Li N., Chen W.-Q. (2021). Changing profiles of cancer burden worldwide and in China: a secondary analysis of the global cancer statistics 2020. *Chinese Medical Journal*.

[7] Pan R., Zhu M., Yu C. (2017). Cancer incidence and mortality: a cohort study in China, 2008–2013. *International Journal of Cancer*.

[8] Eguchi S., Takatsuki M., Hidaka M. (2010). Predictor for histological microvascular invasion of hepatocellular carcinoma: a lesson from 229 consecutive cases of curative liver resection. *World Journal of Surgery*.

[9] Espiritu P. N., Sverrisson E. F., Sexton W. J. (2014). Effect of tumor size on recurrence-free survival of upper tract urothelial carcinoma following surgical resection. *Urologic Oncology*.

[10] Cai M. Y., Wang F. W., Li C. P. (2016). Prognostic factors affecting postoperative survival of patients with solitary small hepatocellular carcinoma. *Chinese Journal of Cancer*.

[11] Kojiro M., Roskams T. (2005). Early hepatocellular carcinoma and dysplastic nodules. *Seminars in Liver Disease*.

[12] Van Waarde A., Jager P. L., Ishiwata K., Dierckx R. A., Elsinga P. H. (2016). Comparison of sigma-ligands and metabolic PET tracers for differentiating tumor from inflammation. *Journal of Nuclear Medicine*.

[13] Arii S., Teramoto K., Kawamura T. (2001). Characteristics of recurrent hepatocellular carcinoma in Japan and our surgical experience. *Journal of Hepato-Biliary-Pancreatic Surgery*.

[14] Harrison L. E., Koneru B., Baramipour P. (2003). Locoregional recurrences are frequent after radiofrequency ablation for hepatocellular carcinoma. *Journal of the American College of Surgeons*.

[15] Mulier S., Ni Y., Jamart J., Michel L., Marchal G., Ruers T. (2008). Radiofrequency ablation versus resection for resectable colorectal liver metastases: time for a randomized trial?. *Annals of Surgical Oncology*.

[16] Zytoon A., Ishii H. K., Murakami K. (2007). Recurrence-free survival after radiofrequency ablation of hepatocellular carcinoma. A registry report of the impact of risk factors on outcome. *Japanese Journal of Clinical Oncology*.

[17] Liu Z., Zhou Y., Zhang P., Qin H. (2010). Meta-analysis of the therapeutic effect of hepatectomy versus radiofrequency ablation for the treatment of hepatocellular carcinoma. *Surgical Laparoscopy, Endoscopy & Percutaneous Techniques*.

The article "Application and Evaluation of a 64-Slice CT Three-Dimensional Fusion Technique in the Determination of the Effective Ablation Margin after Radiofrequency Ablation of Hepatocellular Carcinoma" was retracted in 2023. Reasons: unreliable results or conclusions; concerns about the data; concerns about the peer review; concerns about the citations.

[18] Ahn S. J., Lee J. M., Lee D. H. (2017). Real-time US-CT/MR fusion imaging for percutaneous radiofrequency ablation of hepatocellular carcinoma. *Journal of Hepatology*.

[19] Kai L., Zhongzhen S., Rongqin Z. (2012). Evaluation of ablation safety margin of liver cancer by three-dimensional ultrasound-ct image fusion. *Chinese Journal Of Ultrasound Imaging*.

[20] Makino Y., Imai Y., Igura T. (2013). Utility of computed tomography fusion imaging for the evaluation of the ablative margin of radiofrequency ablation for hepatocellular carcinoma and the correlation to local tumor progression. *Hepatology Research*.

[21] Tang H., Tang Y., Hong J., Chen T., Mai C., Jiang P. (2015). A measure to assess the ablative margin using 3D-CT image fusion after radiofrequency ablation of hepatocellular carcinoma. *Hpb the Official Journal of the International Hepato Pancreato Biliary Association*.

[22] Zhu F., Rhim H. (2019). Thermal ablation for hepatocellular carcinoma: what’s new in 2019. *Chinese Clinical Oncology*.

[23] Hocquelet A., Balageas P., Frulio N., Trillaud H. (2015). Aggressive intrasegmental recurrence of periportal hepatocellular carcinoma after radiofrequency ablation: role of ablative technique and heat-sink effect?. *Radiology*.

[24] Yayong H., Yong D., Hanfeng Y. (2011). Imaging evaluation of liver cancer after radiofrequency ablation. *Chinese Journal Of Clinicians*.

[25] Wakai T., Shirai Y., Suda T. (2006). Long-term outcomes of hepatectomyvspercutaneous ablation for treatment of hepatocellular carcinoma ≤4 cm. *World Journal of Gastroenterology*.

[26] Agopian V. G., Harlander-Locke M. P., Markovic D. (2017). Evaluation of patients with hepatocellular carcinomas that do not produce *α*-fetoprotein. *JAMA Surgery*.

[27] Ruzzenente A., De Manzoni G., Molfetta M. (2004). Rapid progression of hepatocellular carcinoma after radiofrequency ablation. *World Journal Of Gastroenterology*.

[28] Tomonari A., Tsuji K., Yamazaki H. (2013). Feasibility of fused imaging for the evaluation of radiofrequency ablative margin for hepatocellular carcinoma. *Hepatology Research*.

[29] Lee J. Y., Choi B. I., Chung Y. E., Kim M. W., Kim S. H., Han J. K. (2012). Clinical value of CT/MR-US fusion imaging for radiofrequency ablation of hepatic nodules. *European Journal of Radiology*.

[30] Nishigori S., Numata K., Irie K., Fukuda H., Chuma M., Maeda S. (2018). Fusion imaging with contrast-enhanced ultrasonography for evaluating the early therapeutic efficacy of radiofrequency ablation for small hypervascular hepatocellular carcinomas with iso-echoic or unclear margins on conventional ultrasonography. *Journal of Medical Ultrasonics*.

The article "Application and Evaluation of a 64-Slice CT Three-Dimensional Fusion Technique in the Determination of the Effective Ablation Margin after Radiofrequency Ablation of Hepatocellular Carcinoma" was retracted in 2023. Reasons: unreliable results or conclusions; concerns about the data; concerns about the peer review; concerns about the citations.

[31] Xu E. J., Lv S. M., Li K. (2018). Immediate evaluation and guidance of liver cancer thermal ablation by three-dimensional ultrasound/contrast-enhanced ultrasound fusion imaging. *International Journal of Hyperthermia*.

